This article has been retracted.

# miR-30a-5p Inhibits Proliferation and Migration of Lung Squamous Cell Carcinoma Cells by Targeting FOXD1

**DOI:** 10.1155/2020/2547902

**Published:** 2020-04-13

**Authors:** Chunhua Chen, Junhua Tang, Shan Xu, Wenxia Zhang, Hanliang Jiang

**Affiliations:** ^1^Department of Pulmonary and Critical Care Medicine, Sir Run Run Shaw Hospital, School of Medicine, Zhejiang University, Hangzhou 310016, China; ^2^Department of Respiratory Medicine, First People's Hospital of Fuyang, Hangzhou 311400, China

## Abstract

**Objective:**

To investigate the mechanism of miR-30a-5p inhibiting proliferation and migration of lung squamous cell carcinoma (LSCC) cells by targeting FOXD1.

**Methods:**

Bioinformatics was used to analyze differentially expressed genes in the TCGA_LUSC database. qRT-PCR was used to detect the expression levels of miR-30a-5p and FOXD1 in human normal lung epithelial cell line and human LSCC cell lines. The protein expression of FOXD1 was detected by western blot. The cell viability and colony formation abilities were examined by CCK-8 and colony formation assays, respectively. Wound healing and Transwell assays were performed to examine the migration and invasion abilities of cells. The targeted binding sites of miR-30a-5p and FOXD1 were predicted by bioinformatics, and dual luciferase assay was used to verify the targeted binding relationship between miR-30a-5p and FOXD1.

**Result:**

miR-30a-5p was downregulated in LSCC tissues and cells, while FOXD1 was highly expressed. Overexpression of miR-30a-5p or silencing FOXD1 inhibited cell viability, colony formation ability, migration, and invasion of LSCC cells. miR-30a-5p inhibited the proliferation and migration of LSCC cells by downregulating the expression of FOXD1.

**Conclusion:**

miR-30a-5p can downregulate the expression of FOXD1 and inhibit the proliferation and migration of LSCC.

## 1. Introduction

Lung cancer is one of the main causes of cancer-related deaths worldwide. Almost 70%-80% of lung cancers are nonsmall cell lung cancers (NSCLC), including squamous cell carcinoma, adenocarcinoma, and large cell carcinoma [1]. Compared with small cell lung cancer, NSCLC is less sensitive to anticancer drugs and radiation therapy. Recently, molecular-targeted therapies of adenocarcinoma (Gefitinib, erlotinib, and crizotinib) have shown significant therapeutic effects with abundant researches [2]. In contrast, targeted therapies for lung squamous cell carcinoma (LSCC) are still immature. Therefore, more novel treatments for LSCC still need to be discovered.

MicroRNAs (miRNAs) are small noncoding RNA molecules (about 22 nucleotides in length) that often inhibit gene expression at the posttranscriptional level. miRNAs play an important role in many biological processes, such as cell proliferation, invasion, migration, and apoptosis [3]. Previous studies have shown that miRNA expression is significantly different in cancer tissues relative to normal tissues. Human cancer classification can be made on the basis of specific expression characteristics [4] to distinguish cancer subtypes which are closely related to prognosis [5]. Mounting evidence suggests that maladjustment of miRNA is relevant to the development of tumors [3]. In the study of tumor miRNAs, miR-30 has been widely regarded as an important miRNA [6]. The miR-30 family contains five different early-maturing miRNA members (miR-30a, miR-30b, miR-30c, miR-30d, and miR-30e), which play different roles in regulating tumorigenesis and metastasis [7]. miR-30a-5p is a member of the miR-30 family and has been reported to be located in genome-vulnerable region of breast and lung cancer (heterozygous loss of 6q13 chromosome) [8, 9]. miR-30a-5p has received more attention because of its important role in various biological and pathological processes, including development, differentiation, autophagy, and apoptosis [10]. Studies have shown that miR-30a-5p expression is significantly downregulated in NSCLC tissues [11]. This study further identified new targets of miR-30a-5p that may play a role in NSCLC.

The FOXD1 gene is located on chromosome 5q12 and encodes a DNA binding protein of 100 amino acids in length. The FOXD1 protein acts as a transcription factor and contains a forkhead domain that binds DNA as a monomer. It also contains two cycles called “winged helix” [12]. In addition, FOXD1 protein also plays a role in a variety of biological processes, including proliferation, invasion, and tumorigenesis [13]. Heul-Nieuwenhuijsen et al. have found that FOXD1 is increased in prostate cancer tissues and is associated with lymph node metastasis [14]. Zhao et al. have reported that FOXD1 promotes cell proliferation and chemoresistance by inducing breast cancer transition from G1 to S phase [15]. Cheng et al. have reported that FOXD1 is significantly upregulated in glioma samples and regulates colony formation and tumorigenic potential of glioma-derived mesenchymal stem-like cells [16]. Nakayama et al. have demonstrated that FOXD1 is overexpressed in human NSCLC, and patients with high FOXD1 expression have a much shorter survival time than patients with low FOXD1 expression [17]. They also have demonstrated that FOXD1 promotes cell growth and metastasis by activating vimentin in NSCLC.

In this study, we explored the targeted relationship between miR-30a-5p and FOXD1 to identify the potential mechanism underlying proliferation and migration of LSCC cell lines and to find out a new targeted therapeutic approach for LSCC.

## 2. Materials and Methods

### 2.1. Bioinformatics Analysis

Gene Expression Quantification and miRNA Expression Quantification profiles were downloaded from the TCGA_LUSC database (http://ualcan.path.uab.edu/cgi-bin/ualcan-res.pl), including 473 tumor tissue samples and 4 normal tissue samples). DESeq2 and edgeR were, respectively, used for differential analysis (∣logFC∣ > 2, padj < 0.05) to identify the differentially expressed genes and miRNAs (DEGs and DEmiRNAs). Target mRNAs for the mature DEmiRNAs were predicted by miRDB, miRTarBase, and TargetScan databases, and then the miRNA-mRNA network map was constructed by taking the intersection of predicted mRNAs and DEmRNAs. KEGG pathway enrichment analysis was conducted to analyze the mRNA of interest.

### 2.2. Cell Cultivation

The human normal lung epithelial cell line BEAS-2B was purchased from the Cell Resource Center of the Shanghai Institutes for Biological Sciences, Chinese Academy of Sciences (No. 3131C0001000200027), and the human LSCC cell lines NCI-H520 (No. 3111C0001CCC000197), SK-MES-1 (No. 3111C0001CCC000262), and NCI-H1703 (No. 3111C0001CCC000353) were purchased from the Cell Resource Center of the Institute of Basic Medical Sciences, Chinese Academy of Medical Sciences. All cell lines were cultured in RPMI-1640 medium (Sigma) containing 10% fetal bovine serum (FBS) (Gibco, NY), 100 U/mL penicillin, and 100 mg/mL streptomycin (Invitrogen, CA) and were placed in an incubator at 37°C with 5% CO_2_. Subsequent experiments were performed as the cells grew to logarithmic phase.

### 2.3. Cell Transfection

Cells were seeded into 24-well plates and transfected with miR-30a-5p mimic, miR-30a-5p inhibitor, or their corresponding negative control (miR-NC) using Lipofectamine™2000 (Invitrogen) according to the manufacturer's instructions. FOXD1 cDNA and two shRNAs (sh-FOXD1-1, sh-FOXD1-2) against FOXD1 and their negative controls were subcloned into pLenti-GIII-UbC lentivirus vector (Sigma-Aldrich, St. Louis, MO, USA). The empty lentivirus vector group was used as a negative control. The target lentivirus packaging vectors were harvested 24 h after transfection. The miR-30a-5p mimic, miR-30a-5p inhibitor, miR-NC, FOXD1 cDNA, shRNA, and their negative control sequences were synthesized by GenePharma Co., LTD. (Shanghai, China). The NCI-H520 cells were planted in a 24-well plate at a density of 5 × 10^4^ cells/well and cultured at 37°C in a humidified incubator containing 5% CO_2_. After reaching 80% coverage, cells were transfected with target plasmids and lentiviral expression vectors using Lipofectamine™2000 (Invitrogen). The interference efficiency was detected by western blot (WB) 48 h after transfection.

### 2.4. Real-Time Quantitative PCR (qRT-PCR)

Total RNA was extracted from frozen tissues using Trizol (Invitrogen) according to the manufacturer's protocol. The cDNA of miR-30a-5p and FOXD1 were synthesized using a reverse transcription system kit (Invitrogen). qRT-PCR was performed on ABI 7900HT (Applied Biosystems, USA). FOXD1 and miR-30a-5p were normalized by using GAPDH and U6 as internal references, respectively. The primers used were shown in Table 1. The difference in relative expression levels of FOXD1 and miR-30a-5p between the control group and the experimental group was compared by the 2^-*ΔΔ*Ct^ method. The experiment was repeated three times.

### 2.5. CCK-8 Method to Observe Cell Proliferation

Cell proliferation ability was determined according to Cell Counting Kit-8 (CCK-8; Dojindo, Kumamoto, Japan). 3 × 10^3^ cells/well were seeded in a 96-well plate with 100 *μ*l medium. At 0 h, 24 h, 48 h, and 72 h, 10 *μ*l/well of CCK-8 reagent was added into the plate, and the cells were then incubated for 4 h at 37°C. Optical density (OD) value was measured at 450 nm using a spectrophotometer (Spectra Max Plus, Molecular Devices, Sunnyvale, USA) at indicated time points, and the experiment was repeated three times.

### 2.6. Colony Formation Assay

Approximately 2 × 10^2^ cells were seeded in 24-well plates and cultured for 2 weeks in RPMI-1640 medium supplemented with 10% FBS. The medium was then removed, and the colonies were washed twice with PBS. Finally, cells were fixed with 4% methanol and stained with Giemsa for 15 min. The number of colonies was counted under an optical microscope, and the experiment was repeated 3 times.

### 2.7. Wound Healing Assay

The cells were seeded in 6-well plates and cultured for 48 h to form a monolayer. The monolayer was then scraped with a 10 *μ*l pipette tip through the center of the well. Cells were gently washed twice with PBS, and the plates were replenished with fresh medium. After regrowing for 24 h, cells were photographed under a microscope (CKX41, Olympus). The scratch width was measured, and the cell migration was evaluated by the wound healing rate. Wound healing rate = (0 h scratch width − 24 h scratch width)/0 h scratch width × 100%. The experiment was repeated three times.

### 2.8. Transwell Invasion Assay

Transwell chambers (Millipore) with Matrigel-coated polycarbonate membranes were used for cell invasion assay. 5 × 10^4^ cells were suspended in 300 *μ*l of RPMI-1640 medium and placed in the upper chamber. The lower chamber was filled with 6 × 10^2^ *μ*l of complete medium containing 10% FBS. After incubation for 48 h at 37°C, the cells on the upper surface of the membrane were removed. While cells invading to the lower surface of the membrane were fixed and stained with 0.1% crystal violet for 30 min. The number of invaded cells from four random fields was counted under a microscope (100×). The experiment was repeated 3 times.

### 2.9. WB

Proteins were obtained after cells were lysed with lysate buffer and then assessed using radioimmunoprecipitation assay (RIPA, Sigma-Aldrich). Protein concentration was determined using a BCA kit (Beyotime, Jiangsu, China). Protein samples were separated by 10% sodium dodecyl sulfate-polyacrylamide gel electrophoresis (SDS-PAGE) (50 *μ*g/lane) and then were transferred onto a polyvinylidene fluoride (PVDF) membrane. Skim milk was used to block the membrane for 2 h at room temperature. The PVDF membrane was then incubated with the primary antibodies overnight at 4°C. The primary antibodies included FOXD1 (ab179940, 1 : 100, Abcam, China) and GAPDH (ab6721, 1 : 2000, Abcam, China). Afterwards, appropriate horseradish peroxidase- (HRP-) labeled secondary goat anti-rabbit IgG (ab181620, 1 : 10000, Abcam, China) was added for incubation. The intensity of the protein bands was quantified using ImageJ software (NIH, USA) and the experiment was repeated 3 times.

### 2.10. Dual Luciferase Assay

To identify the binding probability of miR-30a-5p with FOXD1 3′-UTR, the 3′-UTR of FOXD1 was cloned to psiCHECK luciferase reporter vector (Sangon Co., LTD., Shanghai, China) to construct wild-type (wt) and mutant-type (mut) FOXD1 HEK293T cells were seeded in 48-well plates and cultured for 24 h before transfection. The miR-30a-5p mimic/NC mimic and psiCHECK-FOXD1 wt/mut vectors were then cotransfected into cells. Finally, luciferase activity was measured by a luciferase assay reagent (Promega, Fitchburg, WI, USA). At least three separate experiments were performed.

### 2.11. Statistical Analysis

All data were processed using SPSS 22.0 statistical software (IBM, SPSS, Chicago, IL, USA). The measurement data were expressed as mean ± standard deviation. The difference between the two groups was analyzed by *t* test. The difference among multiple groups was assessed by ANOVA. *P* < 0.05 was considered to be statistically significant.

## 3. Result

### 3.1. miR-30a-5p Is Lowly Expressed While FOXD1 Is Highly Expressed in LSCC

A total of 3009 DEmRNAs (Figure 1(a)) and 143 DEmiRNAs (Figure 1(b)) were obtained using the edgeR differential analysis in TCGA_LUSC database. 33 mature DEmiRNAs were screened by miRTarBase query, and 790 target mRNAs were obtained as predicted by miRDB, miRTarBase, and TargetScan databases. Eventually, 80 mRNAs with targeted binding sites were found by the intersection of 3009 DEmRNAs and 790 predicted mRNAs (Figure 1(c)). It was found that miR-30a, miR-30d, and miR-130b targeted more cancer-related mRNAs by miRNA-mRNA interaction regulatory network. It has been reported that miR-30a-5p plays an important role in regulating various cancers, and its mutual mRNA is closely related to the occurrence and prognosis of cancer [10, 11]. Therefore, we selected miR-30a-5p for subsequent experiments (Figure 1(d)). Survival analysis of miR-30a-5p-associated mRNAs revealed that there was a significant difference in survival upon high and low expression of FOXD1 (Figure 1(e)). In addition, it was showed that miR-30a-5p was lowly expressed in lung cancer tissues, while FOXD1 was highly expressed (Figures 1(f)–1(g)).

qRT-PCR was used to detect the expressions of miR-30a-5p and FOXD1 in human normal lung epithelial cell line BEAS-2B and human LSCC cell lines NCI-H520, SK-MES-1, and NCI-H1703. The results showed (Figures 1(h)–1(i)) that compared with BEAS-2B, miR-30a-5p was significantly downregulated while FOXD1 was significantly upregulated in three LSCC cell lines (*P* < 0.05). The expression of FOXD1 detected by WB in LSCC cell lines was upregulated (Figure 1(j)). Since the FOXD1 level was the highest in the NCI-H520 cell line, the cell line was chosen for subsequent experiments.

### 3.2. miR-30a-5p Overexpression Inhibits Proliferation, Migration, and Invasion of LSCC Cells

To investigate the effects of miR-30a-5p on proliferation, migration, and invasion of LSCC cell lines, NCI-H520 cells were grouped into NC mimic group and miR-30a-5p mimic group. The results of qRT-PCR showed (Figure 2(a)) that compared with the NC mimic group, miR-30a-5p expression was significantly upregulated in the miR-30a-5p mimic group (*P* < 0.05). Then, the cell viability and colony formation abilities of cells were detected by CCK-8 and colony formation assays, respectively. The results exhibited that (Figures 2(b)–2(c)) overexpression of miR-30a-5p decreased the cell viability and the number of colonies (*P* < 0.05). The wound healing and Transwell assays were used to detect the migration and invasion abilities of cells in each group, respectively. It was observed that (Figures 2(d)–2(e)) overexpression of miR-30a-5p inhibited the migration and invasion abilities (*P* < 0.05).

### 3.3. Silencing FOXD1 Inhibits Proliferation, Migration, and Invasion of LSCC Cells

Next, we explored the effects of FOXD1 on proliferation, migration, and invasion of LSCC cells. NCI-H520 cells were grouped into the sh-NC group, sh-FOXD1-1 group, and sh-FOXD1-2 group. The expression of FOXD1 in each group was detected by WB, and the results indicated (Figure 3(a)) that compared with the sh-NC group, the protein expressions of FOXD1 in sh-FOXD1-1 and sh-FOXD1-2 groups were greatly downregulated (*P* < 0.05). sh-FOXD1-2 group with the most significant decrease in FOXD1 expression was used as the sh-FOXD1 group for subsequent interference experiments. Next, the results of CCK-8 and colony formation assays exhibited that (Figures 3(b)–3(c)) silencing FOXD1 reduced the cell viability and the number of colonies (*P* < 0.05). The results of wound healing and Transwell assays displayed that (Figures 3(d)–3(e)) silencing FOXD1 inhibited the migration and invasion abilities (*P* < 0.05).

### 3.4. miR-30a-5p Targeted Inhibits FOXD1 Expression

Targeted binding sites of miR-30a-5p on FOXD1 3′UTR were predicted through the miRTarBase database (http://mirtarbase.mbc.nctu.edu.tw/php/index.php) (Figure 4(a)). At the same time, the dual-luciferase assay was performed for further verification. The results (Figure 4(b)) showed that the luciferase activity of the miR-30a-5p mimic and FOXD1-wt cotransfection group was significantly lower than that of the NC mimic group (*P* < 0.05), whereas for the miR-30a-5p mimic and FOXD1-mut cotransfection group, there was no significant difference (*P* > 0.05), indicating that FOXD1 was a target of miR-30a-5p. Then, qRT-PCR and WB were used to detect the expression of FOXD1 in NC mimic group, miR-30a-5p mimic group, NC inhibitor group, and miR-30a-5p inhibitor group. The results in Figures 4(c)–4(d) suggested that overexpression of miR-30a-5p significantly reduced the mRNA and protein expressions of FOXD1 (*P* < 0.05), while inhibition of miR-30a-5p posed a reverse effect (*P* < 0.05). miR-30a-5p inhibits LSCC cell proliferation and migration by targeting FOXD1.

The NCI-H520 cells were grouped into NC mimic+oe-NC group, miR-30a-5p mimic+oe-NC group, and miR-30a-5p mimic+oe-FOXD1 group to analyze the effects of miR-30a-5p on the proliferation and migration of LSCC cells by targeted regulating FOXD1 expression. The expressions of miR-30a-5p and FOXD1 in each group were detected by qRT-PCR and WB, and the results showed (Figures 5(a)–5(b)) that compared with NC mimic+oe-NC group, the mRNA and protein expressions of FOXD1 in miR-30a-5p mimic+oe-NC group were significantly downregulated (*P* < 0.05), while, that in miR-30a-5p mimic+oe-FOXD1 group was significantly upregulated compared with miR-30a-5p mimic+oe-NC group (*P* < 0.05). The results of CCK-8 and colony formation assays suggested that (Figures 5(c)–5(d)) compared with the NC mimic+oe-NC group, the cell viability and the number of colonies of the miR-30a-5p mimic+oe-NC group were significantly decreased (*P* < 0.05), while compared with the miR-30a-5p mimic+oe-NC group, those of the miR-30a-5p mimic+oe-FOXD1 group were significantly increased (*P* < 0.05). The results of wound healing and Transwell assays showed that (Figures 5(e)–5(f)) compared with the NC mimic+oe-NC group, the miR-30a-5p mimic+oe-NC group showed a great decrease in migration and invasion abilities (*P* < 0.05), while the miR-30a-5p mimic+oe-FOXD1 group had a remarkably higher migration and invasion abilities than the miR-30a-5p mimic+oe-NC group (*P* < 0.05).

## 4. Discussion

miRNAs have been widely accepted as a regulator of human cancer, and they can be used as a cancer promoter or a cancer inhibitor. miR-30a has been found to be one of the downregulated miRNAs in various types of solid tumors. Many studies have proved that the expression level of miR-30a-5p in NSCLC cells and tissues is significantly downregulated compared to that in normal lung cells [18–21], which is consistent with the results of the present study.

miR-30a-5p has been found regulating tumor development by inhibiting oncogenes in various tumors [19, 22, 23], and it can enhance the sensitivity of NSCLC to paclitaxel by targeting BCL-2 expression [24]. Overexpression of miR-30a-5p can also overcome EGFR inhibitor resistance in NSCLC by modulating the PI3K/AKT signaling pathway [25]. In the meantime, it is also possible to mediate cell proliferation, apoptosis, and migration in NSCLC via the p53/miR-30a-5p/SOX4 axis [19]. In addition, miR-30a-5p also functions in NSCLC by interacting with other targets like CD73/NT5E [20]. This study found that miR-30a-5p directly inhibited the expression of FOXD1. The expression levels of miR-30a-5p and FOXD1 were negatively correlated in LSCC cell lines and normal lung cells. In this study, we performed an online prediction for access of miRNA targets and found possible binding sites within miR-30a-5p and 3′-UTR of FOXD1. The luciferase reporter gene assay results also confirmed the targeted relationship between miR-30a-5p and FOXD1.

A previous study used a microarray dataset including 90 lung cancer specimens to analyze FOXD1 mRNA levels to find that abnormal FOXD1 mRNA was associated with the survival of NSCLC patients. It also reported that knockdown of FOXD1 led to inhibition of cell proliferation, suggesting that the expression of FOXD1 could be used as a novel prognostic factor for NSCLC [17]. In addition, it has been reported that FOXD1 promotes its carcinogenic characteristics by activating Vimentin expression in NSCLC [26]. In this study, we silenced FOXD1 and discovered that the proliferation, migration, and invasion capacities of LSCC cells were inhibited, which was consistent with previous studies. It was also verified that FOXD1 had important research significance for lung cancer.

Traditional treatments for LSCC are radiotherapy, chemotherapy, and lobectomy, which are harmful to patients and have a high risk of side effects and recurrence [27]. Our study confirmed the binding relationship between miR-30a-5p and FOXD1 and found that miR-30a-5p may inhibit the proliferation and migration of LSCC cells by inhibiting FOXD1 expression, which provides new insight into the treatment of LSCC.

## Figures and Tables

**Figure 1:** Expression of miR-30a-5p and FOXD1 in LSCC. Volcano plot of DEmiRNAs (a) and DEmRNAs (b) in TCGA-LUSC; (c) Venn diagram of DEmRNAs and predicted target genes; (d) miRNA-mRNA regulatory network; (e) survival curves of FOXD1 gene. The abscissa indicates the time (years), the ordinate indicates survival rate, the red curve indicates high expression, the blue curve indicates low expression, and each vertical node indicates death of a follow-up individual; relative expression level of miR-30a-5p (f) and FOXD1 (g) in the normal group and the tumor group in TCGA-LUSC; The expressions of miR-30a-5p (h) and FOXD1 mRNA (i) in human normal lung epithelial cell line and human LSCC cell lines were detected by qRT-PCR; (j) The protein expressions of FOXD1 in human normal lung epithelial cell line and human LSCC cell lines were detected by WB. ^∗^*P* < 0.05.

**Figure 2:** miR-30a-5p overexpression inhibits proliferation, migration, and invasion of LSCC cells. (a) The expression of miR-30a-5p in cells transfected with miR-30a-5p mimic and NC mimic was detected by qRT-PCR; Cell viability (b) and colony formation ability (c) of cells in each group were measured by CCK-8 and colony formation assays; The migration (d) and invasion (e) abilities of each group were detected by wound healing and Transwell (100×) assays. ^∗^*P* < 0.05.

**Figure 3:** Silencing FOXD1 inhibits the proliferation and migration of LSCC cells. (a) FOXD1 interference efficiency was detected in cells with miR-30a-5p mimic and NC mimic by WB; The cell viability (b) and colony formation ability (c) of each group were detected by CCK-8 and colony formation assay; The migration (d) and invasion (e) abilities of each group were detected by wound healing and Transwell (100×) assays. ^∗^*P* < 0.05.

**Figure 4:** miR-30a-5p targeted inhibits FOXD1 expression. (a) Targeted binding sites of miR-30a-5p and FOXD1 were predicted by bioinformatics; (b) Targeted binding relationship of miR-30a-5p with FOXD1 was verified by dual luciferase assay; The mRNA (c) and protein (d) expressions of FOXD1 were detected in cells with miR-30a-5p mimic/inhibitor and NC mimic/inhibitor by qRT-PCR and WB, respectively. ^∗^*P* < 0.05.

**Figure 5:** miR-30a-5p inhibits proliferation and migration of LSCC cells by targeted downregulating FOXD1 expression. Relative expressions of miR-30a-5p and FOXD1 in each treatment group were detected by qRT-PCR (a) and WB (b), respectively; The cell viability (c) and colony formation ability (d) of each group were detected by CCK-8 and colony formation assays; The migration (e) and invasion (f) abilities of each group were detected by wound healing and Transwell (100×) assays; ^∗^*P* < 0.05; oe-NC+NC mimic indicates negative control; miR-30a-5p mimic+oe-NC indicates overexpression of miR-30a-5p alone; miR-30a-5p mimic+oe- FOXD1 indicates simultaneous overexpression of miR-30a-5p and FOXD1.

**Table 1:** Primer sequences.

Gene	Primer sequences
miR-30a-5p	F: GGGCCTGTAAACATCCTCG
	R: GAATACCTCGGACCCTGC′

U6	F: GGTCGGGCAGGAAAGAGGGC
	R: GCTAATCTTCTCTGTATCGTTCC

FOXD1	F: AAGAACCCGCTGGTGAAG
	R: GTCCAGTAGTTGCCCTTGC

GAPDH	F: ACAACTTTGGTATCGTGGAAGG
	R: GCCATCACGCCACAGTTTC

## Data Availability

The data and materials in the current study are available from the corresponding author on reasonable request.
